This article has been retracted.

# Additional Acupuncture Confers a Favorable Long-Term Prognosis for Elderly Hypertensive Patients with Carotid Atherosclerosis after Atorvastatin Treatment

**DOI:** 10.1155/2022/7479416

**Published:** 2022-05-16

**Authors:** Jiefang Li, Dan Wu, Jun Liu, Xi Li

**Affiliations:** Traditional Chinese Medicine Department, The Fourth Hospital of Changsha, Changsha, China

## Abstract

**Objective:**

The purpose of the study is to investigate the clinical efficacy and long-term prognosis of acupuncture (AP) combined with atorvastatin (ATO) in treating senile essential hypertension (EH) complicated with carotid atherosclerosis (CA).

**Methods:**

108 elderly EH patients with CA admitted to our hospital between January 2018 and September 2018 were enrolled into the study, consisting of 67 patients who received treatment of AP with ATO (AP + ATO group) and 41 patients who received treatment of ATO alone (ATO group). Comparative outcomes included clinical efficacy, blood pressure (BP), the levels of blood lipids and inflammatory factors, carotid intima-media thickness (IMT), the number of unstable carotid intima plaques, the carotid plaque area, and the incidence of adverse reactions. All patients were followed up for 3 years to evaluate their quality of life and the recurrence rate of CA.

**Results:**

The AP + ATO group presented a higher efficacy, a declined BP, and lower posttreatment levels of blood lipids and inflammatory factors than the ATO group (*P* < 0.05). Reductions were observed in IMT, number of plaques, and plaque area in both groups after treatment, with more significant improvements in the AP + ATO group (*P* < 0.05). No difference was observed in the incidence of adverse reactions between two groups after treatment (*P* > 0.05). The follow-up analysis demonstrated a higher SF-36 score and a lower recurrence rate of CA in the AP + ATO group than the ATO group (*P* < 0.05).

**Conclusion:**

The findings suggested that, for elderly EH patients with CA, treatment of AP with ATO offers better clinical efficacy and safety, which not only can decline the BP, but also can reduce blood lipids and plaque formation, and improve quality of life.

## 1. Introduction

Essential hypertension (EH) is a chronic and common condition in the elderly and middle-aged, which is defined as a condition in which the pressure of blood flowing through the blood vessels continues to be higher than normal, resulting in elevated incidence of cardio-cerebrovascular diseases (CCVDs) and kidney diseases [1]. In recent years, the prevalence of EH has increased with the aging of China's population. Statistics show that by 2030, the cumulative number of EH patients worldwide will exceed 300 million, becoming the disease with the highest number of patients [2]. At present, the pathogenesis of EH has yet to be defined, but the more we talk about its risk factors, involving genetic factors, age, unhealthy lifestyle, etc. The more risk factors gather, the greater the risk of EH [3]. Typical symptoms of EH include headache, fatigue, uneasiness, arrhythmia, palpitation, and tinnitus. At the same time, EH is also the main inducing factor of many major diseases, of which carotid atherosclerosis (CA) is a common comorbidity [4]. Due to the absence of significant symptoms in the early stage of the disease, most patients have plaques when diagnosed, resulting in vascular stenosis or local thrombosis, which easily leads to limb and language disorders [5]. Therefore, the diagnosis and treatment of senile EH complicated with CA are particularly important in clinic.

Atorvastatin (ATO) is a commonly used drug for clinical prevention of CCVDs, which has pleiotropic effects such as enhancing vascular endothelial function, improving blood lipids, as well as anti-inflammation and anti-oxidation [6]. It has now been clinically confirmed to be applicable to the treatment of EH complicated with CA with certain positive effects. For example, the research by authors Pi S et al. demonstrates that ATO can validly reduce the degree of CA and stabilize the blood pressure (BP) changes of patients [7]. However, in the long treatment cycle, the drug resistance and toxic side effects resulting from continuous drug use may affect the therapeutic effect of EH complicated with CA or even cause more serious complications [8]. Hence, the treatment of chronic diseases with application of traditional Chinese medicine (TCM) has gradually received clinical attention. Many scholars have pointed out that acupuncture (AP) has significant clinical treatment for restoring nerve function, improving brain blood supply, dilating brain blood vessels, and improving blood circulation ability, with encouraging therapeutic effects for CA [9, 10]. However, there is still a lack of clinical support for specific standardized operation guidelines. In this study, we investigated the clinical efficacy and long-term prognosis of AP combined with ATO in treating elderly EH complicated with CA.

## 2. Data and Methods

### 2.1. Patient Data

After receiving the approval of the Ethics Committee of our hospital, 108 elderly EH patients with CA admitted to our hospital from January 2018 to September 2018 were selected as participants. Of them, 67 patients receiving AP and ATO treatments were allocated to the AP + ATO group, and 41 patients treated by ATO alone were assigned to the ATO group. Inclusion criteria were as follows: (1) hypertension was recorded as having the previous history of hypertension or systolic blood pressure equal to or higher than 140 mmHg and/or diastolic blood pressure equal to or higher than 90 mmHg for two times in the quiet condition, and CA was confirmed by carotid magnetic resonance (MR) images; (2) complete medical records; and (3) included patients must sign a written consent form. Exclusion criteria were as follows: (1) previous history of malignant tumors; (2) abnormal liver and kidney function; (3) previous history of hyperlipidemia and autoimmune diseases; (4) mental illness, language and communication barriers, and low treatment compliance; (5) chronic infectious diseases; and (6) drug contraindications.

### 2.2. Methods

Patients in both groups were informed by nurses of reasonable daily diet, standardized exercise, real-time monitoring of BP, etc. ATO group was given 10 mg ATO (Beijing Jialin Pharmaceutical Co., Ltd., SFDA Approval No. H19990258), once daily. The patients in the AP + ATO group were additionally given AP treatment, with the acupoints selected referring to the “National Standard of the People's Republic of China-Location of Points.” Patients were placed in the supine position, and acupoints such as Zusanli, Fengchi, Fenglong, Renying, Neiguan, Yanglingquan, and Baihui were routinely disinfected. The depth of needle insertion was determined by the patient's body size. When performing AP at Renying, the carotid artery was moved laterally to avoid being needled. The AP lasted for 25–30 min, and the AP points were pressed for 3–5 min after needling. In both groups, the medication continued for 3 months, while AP therapy implemented in AP + ATO group was conducted twice a week for 12 weeks, with an interval of 3 days.

### 2.3. Blood Collection and Laboratory Detection

Before and after treatment, 5 mL of fasting venous peripheral blood of patients in the two groups was extracted into procoagulant tubes, which were then left standing at ambient temperature for 30 min and centrifuged to obtain serum. One part of the serum was used for the detection of total cholesterol (TC), triglyceride (TG), as well as high- and low-density lipoprotein cholesterol (HDL-C/LDL-C) with the use of an automatic biochemical analyzer. Another part went to the determination of high-sensitivity C-reactive protein (hs-CRP), tumor necrosis factor (TNF)-*α*, and matrix metalloproteinase-9 (MMP-9) using ELISA kits all supplied by Beijing Solarbio Science & Technology Co, Ltd.

### 2.4. Follow-Up

After discharge from hospital, all patients were followed up for 3 years via telephone notification of hospital review with an interval of no more than 6 months. At the last follow-up, patients were scored for their quality of life (QoL) by the health measurement instrument SF-36 from the following eight areas: bodily pain score, vitality, mental health, social function, physical function, role-physical, role-emotional, and general health. Higher scores correspond to better QoL. In addition, CA relapse was recorded during the 3-year prognosis ((IMT > 1 mm) is judged as recurrence), and the recurrence rate was calculated.

### 2.5. Evaluation of Clinical Efficacy and Safety

Crouse plaque scores [11] were used to evaluate clinical efficacy. Markedly effective corresponds to a decrease in the plaque, soft plaque, or ulcered score by over 50% after treatment, with the BP < 140/90 mmHg; if the decrease of the plaque, soft plaque, or ulcered score was ≤ 50% after treatment, with the systolic blood pressure (SBP) decrease ≥ 10 mmHg, it was considered effective. No significant improvement in all indexes and failure to meet the above standards was considered invalid. The response rate was calculated as the number of markedly effective and effective cases among all the cases. The degree of carotid artery stenosis was determined through detecting carotid intima-media thickness (IMT), number of unstable carotid intima plaques, and carotid plaque area using color Doppler ultrasonography. The incidence of adverse reactions including nausea and vomiting, diarrhea, fatigue, dizziness, myalgia, and other events during treatment was recorded to evaluate clinical safety.

### 2.6. Data Analysis

Count data were presented as frequencies or percentages. Numerical data in normal distribution were expressed as mean ± standard deviation. Statistical analysis was performed by SPSS 23.0 software (IBM, Armonk, New York, USA) using independent *t* test, paired *t* test, or chi-square test according to data presentation. Differences were demonstrated to be significant with *P* < 0.05.

## 3. Results

### 3.1. Demographic Variables

Two cohorts of patients were compared with regard to their age, BMI, gender, disease duration, residence, smoking status, drinking status, family history, and nationality. It was found that patients in the AP + ATO group and ATO group showed no significant difference in their age, BMI, gender, disease duration, residence, smoking status, drinking status, family history, and nationality, suggesting that two cohorts of patients were comparable (*P* > 0.05; Table 1).

### 3.2. Additional Acupuncture to ATO Treatment Increased Clinical Efficacy and Safety

The overall response rate was higher in the AP + ATO group (97.01%) than in the ATO group (85.37%) (*P* < 0.05, Table 2). The comparison of adverse reaction incidence after treatment revealed an incidence of 4.48% in AP + ATO group and 14.63% in ATO group, showing no statistical significance between groups (*P* > 0.05; Table 3).

### 3.3. Additional Acupuncture to ATO Treatment Reduced the BP

When comparing the changes of SBP and DBP between AP + ATO group and ATO group, we found no notable difference in BP between AP + ATO group and ATO group before treatment (*P* > 0.05), while a decreased BP was observed in two groups after treatment (*P* < 0.05), with a more significant reduction in the AP + ATO group (*P* < 0.05; Figure 1).

### 3.4. Additional Acupuncture to ATO Treatment Reduced Blood Lipids and Plaque Formation

No distinct difference was observed in blood lipid levels between groups prior to treatment. However, TC, TG, and LDL-C levels decreased and HDL-C increased in both groups after treatment (*P* < 0.05), with more significant changes in AP + ATO group compared with ATO group (*P* < 0.05; Figure 2). After comparing the degree of carotid stenosis, we found that there was no difference in carotid stenosis degree between groups before treatment (*P* > 0.05). After treatment, the IMT, the number of unstable carotid intima plaques, and the area of carotid plaque decreased (*P* < 0.05), with more obvious reductions in AP + ATO group (*P* < 0.05; Figure 3).

### 3.5. Additional Acupuncture to ATO Treatment Attenuated Inflammatory Response

It was found that pretreatment levels of hs-CRP, TNF-*α*, and MMP-9 exhibited no evident differences between AP + ATO group and ATO group (*P* > 0.05). However, their posttreatment levels were all decreased significantly, and the levels in the AP + ATO group were lower than that in the ATO group (*P* < 0.05; Figure 4).

### 3.6. Additional Acupuncture to ATO Treatment Provided a Better QoL

During the 3 years of follow-up, 64 cases in AP + ATO group and 40 cases in ATO group were successfully followed up, with a follow-up rate of 96.30%. The intergroup comparison of SF-36 scores after treatment showed that the scores of all domains in AP + ATO group were higher than those in ATO group (*P* > 0.05). Moreover, posttreatment relapse was observed in 12 patients in AP + ATO group and 11 patients in ATO group, with a total recurrence rate of 18.75% and 27.50%, respectively. The recurrence rate of CA was lower in the AP + ATO group than in the ATO group (*P* < 0.05; Figure 5).

## 4. Discussion

EH is one of the most prevalent chronic diseases among the elderly, with a growing incidence in such patients [12]. EH can cause a series of CCVDs, among which CA is the most commonly seen comorbidity [13]. In the treatment of EH patients with CA, relieving angiosclerosis is the key, while halting the rise of BP is the basis [14]. AP, as one of the most representative treatment methods in TCM, is excellent in its safety and stability, which is very suitable for chronic diseases requiring a long treatment cycle. Therefore, this study has important clinical reference significance by exploring the clinical and prognostic effects of AP + ATO in the treatment of EH complicated with CA.

In order to ensure the reliability and rigor of the experimental results, we first compared patients' clinical baseline data between the two cohorts and found no distinct difference, indicating that there was comparability between the two groups of subjects included in this research. Subsequently, the investigation results of clinical efficacy showed a higher response rate in AP + ATO group compared with ATO group, suggesting that AP + ATO has a more significant therapeutic effect on CA. Yu Y, et al. also pointed out that AP has a certain improvement effect on cerebral thrombosis [15], which can also corroborate the results of this experiment and once again demonstrate the excellent application potential of AP in CA treatment. Furthermore, when comparing the changes of BP and blood lipids, we found that the BP improvement of patients in the study group was more significant, which also shows that AP + ATO is more suitable for EH patients with CA. ATO, one of the most commonly used drugs for regulating blood glucose and blood lipids in clinical practice, can reduce cholesterol synthesis, increase LDL receptor synthesis, and reduce blood cholesterol and LDL-C levels [16]. The protein binding rate of ATO is about 98%, most of which are excreted in the bile in the form of metabolites, with relatively stable drug safety. However, after prolonged use, some patients may experience gastrointestinal reactions of different degrees and even a certain risk of renal failure [17]. Therefore, ATO should be used following the doctor's advice, and strict attention should be paid to the dosage and time of use to ensure drug safety. However, it is well known that the treatment of EH and CA is usually a long-lasting process, and the use of drugs can only achieve disease relief and control, without a clinical cure for EH at present [18]. The limitations of ATO, as we mentioned above, are therefore gradually exposed; that is, there may be varying degrees of drug resistance due to individual differences among patients, as well as increased toxicity caused by excessive accumulation of drugs in the body.

In TCM, CA is considered to be blood paralysis caused by physical deficiency and dysfunction of heart and blood vessels, and its treatment principle lies in dredging chemotherapeutic obstruction of blood vessels and keeping the patency of blood vessels. Therefore, in the AP treatment of CA, AP and moxibustion are usually carried out at Zusanli, Fengchi, Fenglong, Renying, and other points that can promote smooth blood flow [19]. In previous studies, the effect of AP at Zusanli and Fengchi acupoints on the patency and normal operation of vascular function has been verified [20]. Xie Z et al. also found that AP at Renying acupoint can not only lower BP and lipids, but also play a calming and sedative effect, relieving the tension and discomfort of patients [21]. Therefore, in this study, AP was used in addition to ATO, achieving more significant effects. When comparing the degree of carotid artery stenosis and plaques before and after treatment, we found that IMT, number of unstable plaques, and carotid plaque area in patients in AP + ATO group decreased more significantly after treatment. Previous studies have pointed out that vascular compliance in CA patients is generally poor, which also leads to low toughness of arterial blood vessels and a significant decline in smooth muscle contractility, resulting in inflammatory injury and stress response under the impact of blood flow [22]. The application of AP therapy can improve the elasticity of blood vessels and stimulate the activity of endothelial cells, which not only promotes the patency of blood vessels and ensures the normal operation of hemodynamics, but also reduces the occurrence of intravascular injuries and the possibility of plaque formation in arteries [9]. This can also be confirmed by the detection results of inflammatory factors before and after treatment in the two groups. Besides, we found no significant difference in the intergroup comparison of ARs, which also shows that AP with ATO has excellent safety. Furthermore, the actual incidence of ARs in AP + ATO group was determined to be only 4.48%, compared with 14.63% in ATO group. We believe that this may be due to the accelerated operation of the overall metabolic function in patients during AP, which reduces the deposition of ATO in the body and consumes more residual substances in the metabolic cycle, thus lowering the possibility of toxic and side effects. However, this needs further confirmation as the metabolic capacity of patients has not been investigated in this study. Besides, the statistical comparison of the incidence of ARs between the two cohorts may also be accidental due to the small number of patients enrolled, which we will also conduct supplementary studies in follow-up experiments.

Finally, in the follow-up of prognosis, we found significantly higher prognostic QoL in AP + ATO group. And the comparison of disease recurrence rate also identified a lower recurrence rate of CA in AP + ATO group, suggesting that AP + ATO can improve the condition of EH patients complicated with CA in a stable and long-term way, and enhance their prognosis, which has higher clinical application value. Moreover, AP and moxibustion treatment of TCM is cost-effective and will not cause great economic burden to patients in the long run, so it is worth popularizing to grassroots hospitals to provide more effective treatment guarantee for the majority of EH patients with CA.

This study has several limitations needed to be elucidated. First, due to retrospective nature, a smaller sample size, and absence of carotid vessel wall imaging during follow-up, future studies with a larger sample size and using 3D vessel wall imaging techniques with larger longitudinal coverage are required.

In conclusion, additional acupuncture to ATO treatment offers better clinical efficacy and safety, which not only can decline the BP, but also can reduce blood lipids and plaque formation, and improve quality of life of elderly EH patients with CA.

## Figures and Tables

**Figure 1:** Blood pressure changes before and after treatment. (a)SBP before and after treatment; (b) DBP before and after treatment. *Note.*^*∗*^ indicates *P* < 0.05 compared with pretreatment level, and & indicates *P* < 0.05 compared with the AP + ATO group.

**Figure 2:** Blood lipid levels before and after treatment. (a) TC before and after treatment; (b) TG before and after treatment. (c) HDL-C before and after treatment; (d) LDL-C before and after treatment. *Note.*^*∗*^ indicates *P* < 0.05 compared with pretreatment level, and & indicates *P* < 0.05 compared with the AP + ATO group.

**Figure 3:** Changes of carotid stenosis degree before and after treatment. (a) Changes of IMT before and after treatment; (b) changes in the number of unstable carotid intimal plaques before and after treatment; (c) changes of carotid plaque area before and after treatment. *Note.*^*∗*^ indicates *P* < 0.05 compared with pretreatment level, and & indicates *P* < 0.05 compared with the AP + ATO group.

**Figure 4:** Comparison of inflammatory factors before and after treatment. (a) hs-CRP before and after treatment; (b) TNF-*α* before and after treatment; (c) MMP-9 before and after treatment; (d) LDL-C before and after treatment. *Note.*^*∗*^ indicates *P* < 0.05 compared with pretreatment level, and & indicates *P* < 0.05 compared with the AP + ATO group.

**Figure 5:** Comparison of quality of life. (a) Bodily pain score; (b) vitality score; (c) mental health score; (d) social function score; (e) physical function score; (f) pole-physical score; (g) role-emotional score; (h) general health score; (i) CA recurrence rate. *Note.*^*∗*^*P* < 0.05.

**Table 1:** Comparison of baseline data between two groups.

	AP + ATO group (*n* = 67)	ATO group (*n* = 41)	t or *χ*^2^	*P*
Age	68.1 ± 4.6	68.0 ± 4.0	0.115	0.909
BMI (kg/cm^2^)	25.87 ± 1.86	25.18 ± 1.87	1.867	0.065
Gender			0.473	0.492
Male	38 (56.72)	26 (63.41)		
Female	29 (43.28)	15 (36.59)		
Disease duration (years)	5.18 ± 1.08	5.54 ± 1.05	1.699	0.092
Antihypertension treatment	34 (50.75%)	20 (48.78%)	0.198	0.843
Residence			0.091	0.763
Urban	46 (68.66)	27 (65.85)		
Rural	21 (31.34)	14 (34.15)		
Smoking			0.238	0.626
Yes	36 (53.73)	24 (58.54)		
No	31 (46.27)	17 (41.46)		
Drinking			0.409	0.523
Yes	40 (59.70)	27 (65.85)		
No	27 (40.30)	14 (34.15)		
Family history of EH			0.035	0.853
Yes	58 (86.57)	36 (87.80)		
No	9 (13.43)	5 (12.20)		
Nationality			0.391	0.532
Han nationality	64 (95.52)	38 (92.68)		
Minority	3 (4.48)	3 (7.32)		

**Table 2:** Clinical efficacy between the two groups.

	AP + ATO group (*n* = 67)	ATO group (*n* = 41)	*χ* ^2^	*P*
Markedly effective	40 (59.70)	14 (34.15)		
Effective	25 (37.31)	21 (51.22)		
Ineffective	2 (2.99)	6 (14.63)		
Total effective rate (%)	97.01	85.37	5.032	0.025

**Table 3:** Incidence of adverse reactions between the two groups.

	AP + ATO group (*n* = 67)	ATO group (*n* = 41)	*χ* ^2^	*P*
Nausea and vomiting	1 (1.49)	1 (2.44)		
Diarrhea	0 (0.0)	1 (2.44)		
Fatigue and dizziness	1 (1.49)	2 (4.88)		
Myalgia	1 (1.49)	2 (4.88)		
ARs (%)	4.48	14.63	3.435	0.064

## Data Availability

The data used to support the findings of this study are included within the article.
